# Application of CAD in Landscape Grid Space Design and Drawing

**DOI:** 10.1155/2022/5800183

**Published:** 2022-04-25

**Authors:** Shuang Qiao, Yanbin Liu, SuYoung Lee

**Affiliations:** ^1^Mudanjiang Normal University, Mudanjiang 157000, Heilongjiang, China; ^2^Kunsan National University, Gunsan 541150, North Jeolla Province, Republic of Korea

## Abstract

CAD technology has brought great convenience and effect to the design. This paper proposes to update the comparative analysis of the basic classical landscape grid space structure by constructing a landscape grid space design. According to the actual situation of domestic landscape grid space design and drawing, this paper highlights the role of CAD technology in landscape grid space design and drawing and provides an important basis for the subsequent application of CAD software in landscape grid space design.

## 1. Introduction

In the past, the design planning of landscape grid space came from the designers' work experience [1, 2]. If in the face of the planning and design of large landscape grid space [3, 4], we pay special attention to designers' rich experience, design hours, and artistic cultivation [5, 6]. Now, the CAD technology function is becoming more and more mature, and the landscape grid space design planning using CAD technology function design has the advantages such as humanized and intelligent. Compared with previous methods of work experience, CAD technology is more scientific, accurate, and efficient. At present, the design method of CAD technology computing method is becoming more and more mature, and the research design of logic process has become the main direction in this field [7, 8]. Using the parametric method to choose landscape environment gives an important data source.

CAD software has rich graphics library, and landscape doors, windows, some trees, and lawn can be modified by CAD software or can directly call the scheme plan. In addition, you can draw good graphics such as flower stands, drawing planes, and stereoscopic images, such as pavilions and corridors. Put duplicate drawings in the database before it is easy to use. Through the above research data, this paper proposes to use CAD technology in the landscape grid space design planning, landscape road line selection through experiments and is more accurate and efficient than the traditional computing methods.

## 2. Analysis of Spatial Design of Landscape Grid

### 2.1. CAD Software in the Landscape Grid Space Design Application

The source channel of the CAD technology is a two-dimensional planar system. It contains publications, promotional works, images, and maps. Especially in the era of developed science and technology, the static information graphics pattern is still a traditional visual expression, and more innovative factors should still be added to make the creative works of urban landscape grid space culture active. For example, the concept of the Beijing Palace Museum was the background of Emperor Yongzheng in the Qing Dynasty. The innovative fan is according to the static text, and is to simplify the text factors, the form of cultural creative works, material, technology processing, and consumer demand elements, set up the brand image, make consumers from the style of the fan feel the Qing dynasty yongzheng historical development and product characteristics, represent the image of the Qing period, and carry forward the essence of urban landscape grid space culture [9–11].

According to the guidance of the cultural works scheme of Changsha urban landscape grid space, through the static graphics theory, give full play to the charm of Changsha with simple lines and bright colors, display Changsha's famous scenic spots and geographical indications, and let tourists associate and resonate with urban culture [12, 13]. There is no strict gap between the dynamic and static aspects of CAD technology. The CAD technology is capable of transforming the dynamic CAD technology. For example, in the author's world, the creation of dialect cultural masks is based on the landscape grid space. Through the design of garden landscape grid space through word of mouth, CAD technology replaces the mobile dynamic information communication mode. Through creation and expression, we explain the thoughts in dialect in the form of pinyin in dialect and launch interesting dialect learning activities, so as to make learning dialect relaxed and interesting or even convey a feeling. It can let visitors not only experience the interesting landscape grid space life but also enjoy the historical process of Changsha and the customs and life of the local people.

In creation, it is necessary to integrate the preferences of tourists and use the design concept of H5 page to make the local dialect have more cultural atmosphere and personality expression. Use online vivid graphic to make dialect communication more vivid. This is the idea that dialect culture really wants to express and spread, and it is the effect conveyed to tourists at a different level. The dynamic and static information graphics concept can be transformed or even combined with each other, enhancing the permeability and influence of urban cultural communication and making the way of communication wider.

### 2.2. Introducing the CAD Software Design Method

The initial path optimization obtained based on the path design drawing algorithm using CAD being the initial value of the grid space design algorithm. Points S, P1, P2 etc. set the different nodes of the initial path. Pi1 represents the beginning node of the road selection segment, and Pi2 represents the end node of the road selection section, with any point of the segment as follows:

(1) $$\begin{array}{c} P_{i}\left(h_{i}\right)=P_{i1}+\left(P_{i2}-P_{i1}\right)\times h_{i},h_{i}\in \left[0,1\right],i=1,2,\cdots . \end{array}$$

Then, the path length from source point S to end point *T* can be expressed as

(2) $$\begin{array}{c} L=\left\{S,P_{1}\left(h_{1}\right)+\sum_{i=1}^{d-1}length\left\{P_{i}\left(h_{i}\right),P_{i+1}\left(h_{i+1}\right)+P_{d}\left(h_{d}\right)\cdots \right\}\right\}. \end{array}$$

Different combinations can represent pathways of different lengths. Therefore, the problem of finding the best path through the landscape group algorithm is to find a suitable value. Let the number of views of the nest be *R* and the set of elements to be optimized be *D*; *D*_*φ*_*i*__ represents its *i*(1 ≤ *i* ≤ *n*) th element. The variable to be optimized is *h*_1_, *h*_2_, ⋯, *h*_*d*_, and the number is *n*.

(3) $$\begin{array}{c} k\left(\zeta_{j}^{t}\left(D_{\varphi_{i}}\right)\right)=\frac{\zeta_{j}\left(D_{\varphi_{i}}\right)}{\sum_{i=1}^{n}\zeta_{j}\left(D_{\varphi_{i}}\right)}. \end{array}$$

The formula indicates the probability of judging different estimates only by the *t* scenery *k*(*ζ*_*j*_^*t*^(*D*_*φ*_*i*__)).

View search is adjusted to [9]:

(4) $$\begin{array}{c} \zeta_{j}\left(D_{\varphi_{i}}\right)\left(t+\Delta \right)=\zeta_{j}\left(D_{\varphi_{i}}\right)\left(t\right)+\Delta \zeta_{j}\left(D_{\varphi_{i}}\right), \end{array}$$

where Δ*ζ*_*j*_(*D*_*φ*_*i*__) expression represents the total number of remaining information elements of the scenery through all elements *φ*_*i*_. This calculation is made as follows:

(5) $$\begin{array}{c} \Delta \zeta_{j}\left(D_{\varphi_{i}}\right)=\sum_{k}^{R}\Delta \zeta_{j}^{k}\left(D_{\varphi_{i}}\right). \end{array}$$

Repeat the above procedure until the maximum number of iterations allowed or all views obtain a unique element, and then *h*_1_, *h*_2_, ⋯, *h*_*d*_ is the optimized.

Over time, since the exploration process of landscape groups is accompanied by pheromone volatilization, it is necessary to reasonably update the pheromone information on the pathway.

(6) $$\begin{array}{c} \tau_{ij}\left(t+1\right)=\left(1-\rho \right)\tau_{ij}\left(t\right)+\rho \tau_{0}. \end{array}$$

In the formula, *τ*_0_ indicates the initial pheromone concentration. *ρ* indicates the pheromone volatilization coefficient.

The global pheromone update rule is

(7) $$\begin{array}{c} \tau_{ij}\left(t+1\right)=\left(1-\rho \right)\tau_{ij}\left(t\right)+\rho \Delta \tau_{i,j}\left(t\right),\\ \Delta \tau_{i,j}\left(t\right)=\frac{1}{L_{b}}. \end{array}$$

For the CAD software, parameter setting is complex and difficult to start with the shortcomings; you can import the CAD software. This software is simple and can simply model with it. After modeling using the CAD software, some changes occurred in the overall design flow as shown in Figure 1.

### 2.3. Vector Map Software and Bitmap Software Are Introduced

Due to the poor modeling ability of CAD software, the loss of image amplification is often the disadvantage of bitmap software, which can be overcome by vector map software and bitmap software. In the process of drawing the plane plan, first draw the CAD wire frame diagram to color it on this basis to make up for the lack of bitmap software. This is the hand-painted pen, signature pen, pencil, and other linear shape; first, draw the frame of the design map. Use marker, colored lead, watercolor, and other tools to make up for their shortcomings.

### 2.4. Landscape Grid Space Design Is Innovative

In addition to reflecting the rationality, the design of the landscape grid space plan also pays attention to innovation, and certain artistic rules should abide by in the design. One is the relationship between diversity and unity[14]. Diversity refers to the diversification of garden landscape design in terms of design forms and should be rich and varied in terms of dimensions, colors, lines, forms, styles, and other factors. Unity refers to taking the above factors into account, making them unified and coordinated to form a certain degree of similarity or consistency, making people feel that each element in the design does not exist in isolation. Then, I felt messy and unruly. Second, grasp the relationship between coordination and comparison. The design of landscape grid space achieves the purpose of harmony by grasping and innovating the body shape, color, line, proportion, reality, and dark, forming different forms of objects as the whole. It is related to the different scenery. Third, the relationship between balance and stability. Landscape grid space is being designed, and it is necessary to consider color issues. It would be messy if it is thick. The issue of quantity must also be considered. It is too much, just incongruous. According to the principle of balance, only the reasonable combination of the weight of various plants can make it feel stable and comfortable. The fourth is the relationship between rhythm and rhythm. The morphology, color, and texture of the plant can show the rhythm and rhythm of the landscape. Willow needs to be detailed and funny, considering the mood and law, the most suitable for the effect of the landscape. Arrange designed vegetation to enhance the sense of rhythm and rhythm.

The paving of landscape grid space is not the main landscape, but the coordination with unreasonable areas, making each area more clear, shape, and pattern to foil the environment and increase the sense of thickness of landscape grid space. The decoration is more centered on neutral tone, and the color is not vulgar, but generally speaking, luxurious color should be coordinated with the atmosphere of landscape grid space and make use of line of sight and strengthen the sense of direction and openness of space.

Landscape grid space sketch is the decoration after the completion of the landscape grid space construction, through the flower bed lighting appliances, flower rack, chairs, rocks, vegetation, flower bowl, and spring hanging, carving of the ornament to meet people's physiological and psychological requirements. Landscape grid space sketch separates the space contact space, so that each scenic spot has obvious marks. The landscape through the memorial park is exaggerated by the sketch. The overall atmosphere of the landscape garden shows a unique artistic conception, exploration, longing, and other artistic conception.

### 2.5. Rationality of the Garden Landscape Grid Space Design

Landscape grid space plan design has certain ideas, through the whole process of landscape grid space, through the establishment of the idea, grasping the landscape grid space design direction, the design concept into all aspects of the plan, the guiding ideology is the central point of planning design, mastering the leadership thought, and designing to meet the needs of the landscape grid space works. The content of the modern garden landscape grid space design plan is becoming more and more complex. It has something to do with raising people's aesthetic appreciation. To live, living requires a wide variety of activities. In the design, it not only considers people's activities to design but also pays attention to the play of the function. The landscape design of the memorial park is not only limited to quadratic elements but also needs three-dimensional and three-dimensional display environmental space capacity to meet the needs of people's activities.

Scientific and detailed investigation and research always follow the basic principles of landscape grid space planning at home and abroad. This mainly depends on the social reasonable nature of the landscape grid space planning discipline. Through reasonable scientific landscape grid space planning, plan various construction procedures and make effective use of the data collected to understand the public opinion. Through the investigation of local culture and nature, the landscape design of the memorial park can be more scientific and can realize the unity of history and the future. Landscape grid space is complex system engineering, so need scientific and reasonable design drawing, continuous analysis of each system intervention engineering each stage, clear theme, through comprehensive research to solve the problem of investigation, grasp the main contradiction, from the enemy put forward the correct strategic deployment, and make landscape grid space planning design healthily develop along the right direction. In order to commemorate the design plan of the park landscape, the plan needs to be decided according to the comparative law and empirical law. By imagining the future, argumentation will play an important role if seeking new ideas and new ideas.

## 3. Main Functional Analysis of the Engineering Design CAD Software

Landscape grid space planning design is the discipline of dealing with human living space and natural relations. In the historical process, its connotation and extension have changed. The relevant content is not only limited to the traditional pavilions, pavilions, rocks, and wood construction but also included in a larger category. The name of landscape grid space discipline is from garden to landscape grid space, which explains an expansion and inclusion of landscape grid space discipline. In the process of professional landscape grid space, in the garden and garden era, culture and art have emphasized the design core content, from “based in nature, higher than nature” “architectural beauty and natural beauty blend” “poetry interest” to “artistic conception connotation” all not emphasizing the characteristics of garden, rising to the philosophy is the idea of “unity of man and nature”. The core of the garden design of nature is that the focus is to illustrate one. Poetic painting; garden; architecture; and pure design concept often ignore the specific design operations, especially CAD technology design technology.

### 3.1. Library Management

The use of CAD software in the landscape grid space design is relatively complex. In the relevant landscape grid space design, the amount of data and information involved is large, and the types of landscape grid space design are also large. However, in order to better face the landscape grid space design subject, we need to make contact with the landscape grid space design mode. Among them, the landscape grid space design graphics data mainly contain the finalized design drawings needed by the designer to carry out the engineering design. According to some special scattered design drawings compared with the traditional engineering design, CAD software in addition to the most basic data mode processing, I understand the need to handle several text data and data.

CAD software contains standard template library, design parameter library, and design drawing library. Among them, the main role of the standard template database is to save the design roadmap, the main role of the design parameter database is to save the design parameters, and the main role of the design drawing database is to save the engineering drawings. Previous business databases processed data types mainly numbers and text, but engineering classes also contain nonstructured graphics data.

### 3.2. Engineering Management

As the project becomes more and more complex, especially in the field of landscape grid space design, the personnel and professionals involved in the design also show a gradually increasing trend. With the number of relevant designers increasing, the concepts of design and common design are constantly proposed. In addition, there are more projects to design now. In addition, the relevant design has the possibility of revision and change. This allows the CAD software to effectively implement the management of design projects and constantly meet the multivariability of design methods and project changes and modifications. Therefore, during the engineering design, additional engineering management functions will be added to the CAD software. For example, in the spatial design map of the courtyard landscape grid, the addition of the project management function greatly meets the modification and change of the garden landscape grid based on the spatial design.

In the Internet era, information is changing rapidly, and cultural communication is also extensive. Nowadays, the garden landscape grid space cultural creation products need further design and communication services. The graphic theory of information sharing is the publicity background of the website, and the interface design of the mobile phone is also the key content. Now, consumer aesthetic vision and convenient way of pay, using the platform of creative APP communication landscape grid space cultural creative products, using the form of electronic positioning platform and network application, can make the cultural creative products continue late value-added services, help tourists and landscape grid space city both communicate and understand each other. It is the experience of the cultural characteristics of the creative products of urban landscape grid space and the personalized and intelligent landscape grid space happiness brought to tourists. The Internet combines the design of urban landscape grid space and spreads the form of landscape grid space design with a new mode. With the rapid development of economy, the development of landscape grid space design is more challenging and breakthrough.

## 4. Application of CAD in Landscape Grid Space Design and Drawing

CAD rationally allocates road system, building, water body, and plant configuration according to the actual situation, making modification, movement, and direction adjustment, which is consistent with the actual situation to the greatest extent. Garden office building project first according to the general plan and building plan (Figure 2, in cm, level the ground of the construction site, and determine the outdoor zero elevation of 0.000. Line from the site ground. Dig the foundation pit of the positioning axis. Basic engineering: based on the previous 2-D construction drawing 2,3-D structure construction drawing was made, focusing on 3-D structure construction drawing and dynamic observation (combined with dwg documents) to scientifically guide and construct the garden office buildings. The specific construction process is as follows.

### 4.1. Site Point, Discharge, and Excavation Construction of Foundation Pit

Determine and mark the axis pile (200 cm from the foundation pile) while completing the site discharge line on the building plan site. Vertical shaft piles are as follows.  Figure 3 shows the horizontal shaft piles as follows. Point and line the pits intended to dig. In addition, margarine made of lime powder is used, and the depth vertical to the bottom of the building is the foundation of 110 cm. The stairs are based on 62 cm. The width is shown in Figure 3.

### 4.2. Construction of Foundation Beams (Fences) and Columns

After digging out the pit, the bottom of the pit was fixed manually or mechanically, and the gravel and wet sand were first filled together in the pit of the building. The artificial foundation is 15 cm. ThickAdd C20 concrete and stamp firmly. The thickness of the pad is 15 cm. After the pit of the stairs is compacted at the bottom, the vibration of the C20 concrete is applied directly to make it flat. The thickness of the pad is 12 cm. After the concrete is hardened, the central point of the pile shall determine the center of the position of the formwork of the foundation beam with the bullet beam. Install the foundation beam formwork first and then harden the C30 concrete according to the general drawing of the reinforcement structure of the building (building, stairs, and pavilion) (Figure 4) to make it smooth. After the concrete of the foundation beam is hardened, set out to determine the center of the column and the location of the column formwork. First, install the reinforcement of the foundation column, install the formwork, apply the vibration of C30 concrete, and make hard contact. Cover with sacks, maintenance concrete with the fountain (same below), after 8∼30d, and fill earth and sand and complete foundation work (Figure 5).

### 4.3. Construction of Building Posts and Stair Posts

The foundation columns of the building and stairs are on the plane, and the location of the bullet line determines the location of the columns of the building and the columns of the stairs, with construction drawings in 3 *D* (Figure 6). The main line of the building and stairs continue to extend the threaded hill to tie the fixed strap of the column and stairs column, then install the column template with the column hoop (bottom 3 cm and height 6 cm of wood bar specification), support the fixed column template 1/4 around the column template with 4 rods (6 cm diameter), and correctly locate the center point and attached drawings of the column. After correct inspection, pour C40 concrete, clean, and complete the column and stair work (Figure 6).

### 4.4. Construction of Stair Formwork and Reinforcement

After 10–15 d of stair column concrete placement, flatten the floor of the stairs. Set up the scaffolding for the stairs. First install the formwork of the stair platform beam, install the base formwork of the stair and the stair, install the steel bar is fixed with wire, install the formwork of the stair kick, and complete the formwork of the stair and reinforcement (Figure 7).

### 4.5. Construction of Pavilions and Columns

In order to make the column Japanese pillars to connect the column and the main line welding, there is a wind resistance and seismic structure. (40 cm × 40 cm) and pavilion columns (25 cm × 25 cm) because the intermediate backbone muscle bending the column bar to the inside was 17° and 4 angles 24°. Weld the main muscle corresponding to the pavilion column, so that the bottom of the husband muscle contact with the ground. (Figures 8 and 9). After the completion of the concrete pouring floor, 28–30 d, determine the center point of the pavilion and formwork with barbed wire, install the pavilion box with 4 rods at 1/4 of the periphery, confirm the correct installation of reinforcement and type frame, and add C40 to complete the construction of the booth with concrete (Figure 8).

### 4.6. Construction of Pavilion Beams and Pavilion Roof

For pavilion scaffolding, please refer to the installation of scaffolding. First, install the beams of the pavilion and the inclined wall of the roof of the pavilion and then install the formwork of the ceiling. The reinforcement is installed in the same order as the formwork. Verify that the formwork and the reinforcement are installed correctly (Figure 10). C30 concrete pouring is based on injection and maintenance according to the order of mold installation and complete the pavilion beam and roof works.

### 4.7. Demolition of Formwork, Construction of Wall, Pavilion Facilities, and Roof and Stair Railings

The concrete poured in the pavilion passes between 60 and 80 d. After the strength of that concrete reaches the strength, the formwork can be removed. The pavilion mold is the plate under the plate *T* beam on the *T* inclined beam side of the pillar *T*, the stair mold is the plate 5 under the step plate (kick board)—the section side. After removing the formwork, the construction according to the dimensions is shown in the 3 *D* construction drawing (Figure 11) (the exterior wall 18 wall, the height difference of +15 cm, bench 42 cm, width 40 cm, and roof and the stair railing are 83 cm), and the materials complete the construction of the main body of the office building on the 1 floor wall, under the pavilion facilities, the roof armrest and the handrail of the stair, respectively.

Using the above methods can greatly improve work efficiency, avoid labor repetition, shorten the design and planning cycle, and better meet the design needs. However, to cultivate the design, the selection of tree species is inevitable not only meeting the needs of human aesthetic consciousness but also meeting the local growing environment, which is a key problem of the carefully cultivated design in the landscape grid space design plan. For this case, when making the corresponding software, conduct the design and planning. According to the growth environment of the tree species, the applicable area and some basic tree species form information. Reasonable selection of tree species: in addition, the region's climate, soil, in-depth analysis, hydrological understanding, and other information formulates a reasonable planting plan and better meets people's aesthetic needs.

## 5. Conclusions

Application of CAD technology in landscape grid space: we study the design results in CAD grid design and drawing in multimedia environment. Compared with the traditional form, the path length of multimedia environment CAD technology is small and the efficiency is higher. This method can better meet the requirements of garden design and drawing.

## Figures and Tables

**Figure 1:** Design process of landscape grid space optimized by Sketch Up software.

**Figure 2:** Plan of the garden office building.

**Figure 3:** Site point, discharge, and excavation structure of foundation pit.

**Figure 4:** Floor, stairs, and pavilion.

**Figure 5:** Foundation reinforcement and formwork structure.

**Figure 6:** Reinforcement and formwork structure of building columns and stair columns.

**Figure 7:** Stair scaffold, formwork, and steel structure.

**Figure 8:** Steel bar amplification structure of the pavilion.

**Figure 9:** Bar and column reinforcement and formwork structure.

**Figure 10:** Pavilion beam and roof scaffolding, formwork, and reinforcement structure.

**Figure 11:** Effect of garden office building (aboveground and + underground).

## Data Availability

The labeled dataset used to support the findings of this study are available from the corresponding author upon request.
